The article "Application of LSTM algorithm combined with Kalman filter and SOGI in phase-locked technology of aviation variable frequency power supply" was retracted in 2023. Reasons: unreliable results or conclusions; concerns about the results or conclusions; concerns about the peer review.

# Application of LSTM algorithm combined with Kalman filter and SOGI in phase-locked technology of aviation variable frequency power supply

**DOI:** 10.1371/journal.pone.0263634

**Published:** 2022-04-14

**Authors:** Bo Zeng, Yuxiang Sun, Shaojun Xie

**Affiliations:** 1 College of Automation Engineering, Nanjing University of Aeronautics and Astronautics, Nanjing City, China; 2 School of Management & Engineering, Nanjing University, Nanjing City, China; 3 School of Computing and Engineering, University of Derby, Derby City, United Kingdom; Ministry of Natural Resources North Sea Bureau, CHINA

## Abstract

With the development of computer technology, the concept of computer automatic control has gradually penetrated the research field of aircraft power control, and intelligent power control systems have become mainstream research. The present work aims to improve the performance of the broadband phase-locked loop (PLL) based on the linear Kalman filter. Specifically, this paper first introduces linear Kalman filter and second-order generalized integrator (SOGI). Then, SOGI is added to PLL based on the linear Kalman filter. The purpose is to use the infinite gain effect of SOGI at the central angular frequency to eliminate the time-varying angular frequency component in the error when the system inputs SOGI to achieve a better filtering effect. Then, the system’s stability analysis and parameter settings are carried out to establish an intelligent phase-locked method of aviation variable frequency power supply. Finally, simulation experiments are performed. The experimental results demonstrate that PLL via the linear Kalman filter with SOGI can solve the problem that the output phase angle contains high-frequency components when the power supply voltage distortion rate is 10%. This scheme has a strong anti-interference ability under power grid voltage imbalance. The accuracy of the Long and Short-term Memory network used here is about 80%, which can well realize the intelligent aviation power frequency conversion control method. The research reported here provides a reference for establishing smart phase-locked technology of aviation variable frequency power supply.

## 1 Introduction

As the multi-electric aircraft technology constantly advances, the aircraft power system capacity increases, realizing higher power generation efficiency. The advantages of aviation variable frequency power supply without constant installation and converter are gradually emerging [1–3]. The three-phase rectifier is a critical power conversion link in airborne electrical equipment. The high-power factor is one of the fundamental indexes to measure the performance of rectifiers for aviation applications. It is necessary to obtain grid voltage phase information to achieve high power factor operation of the rectifier, which is usually completed by a phase-locked loop (PLL). The wide operating frequency range (typically 360-800Hz) of aviation variable frequency power supply and the characteristics of small capacity grid voltage easily affected by load distortion put forward higher requirements for phase-locked technology on this occasion. The requirements for the phase-locked technology of high-power factor rectifier power supply of the system are increasing due to the particularity of the frequency range of aviation variable frequency power supply and the problem that the load easily distorts the power supply voltage. Many pieces of literature have studied the phase-locked technology of aviation variable frequency power supply with a wide working frequency range and less harmonic content. A second-order generalized integrator (SOGI) is added in the front stage of PLL to realize accurate phase locking in the environment of the high harmonic range of power supply voltage and unbalanced three-phase grid voltage. SOGI is a typical second-order filter that simultaneously generates two mutually orthogonal signals. Besides, its transfer function has infinite gain in a specific frequency.

Reference [4] proposes a PLL based on the discrete Fourier transform (DFT) algorithm for aviation variable frequency power supply systems. Its principle is to separate the fundamental component of the power supply by using the DFT algorithm and then use Proportional Integral Controller as a loop filter. Finally, a PLL is completed by corresponding calculation. However, the dynamic response is slow due to the algorithm’s complexity, and the phase information cannot be obtained quickly. A PLL of Steady-state linear Kalman filter (SSLKF) is put forward in references [5, 6], an adaptive phase-frequency estimation algorithm based on a third-order linear constant observation model and a predictive correction model. Three different control units are used to estimate phase angle, angular frequency, and angular frequency acceleration, respectively, with high phase-locked accuracy, fast dynamic response, and other advantages. In reference [7], two PLLs are comprehensively compared in dynamic performance, phase-locked accuracy, and filtering effect. It is concluded that the linear Kalman filter PLL has more advantages. Therefore, the linear Kalman filter PLL is more suitable for the phase-locked system of aviation variable frequency power supply. However, the phase-locked technology of aviation variable frequency power supply with high harmonic content has not been studied in the existing literature. According to the DO-160G standard, the maximum single voltage distortion rate of aviation variable frequency power supply is 8%, and the maximum total voltage distortion rate is 10%. The linear Kalman filter PLL is applied to the environment with a low power supply voltage distortion rate. Although good phase-locked results are obtained, when the distortion rate of aviation variable frequency power supply reaches 10%, the output phase angle of linear Kalman filter PLL contains high-frequency components, which affects the overall performance of the converter. In references [8–11], the convergence of differential equations solutions is used to judge the system’s stability, which concerns the analysis of high-order nonlinear systems. Inspired by the method proposed in reference [12], this paper presents the structure of linear Kalman filter PLL with SOGI. Most of the PLLs in the existing literature are applied to the linear analysis of the small-signal model. There is a significant deviation from the linear model of small signals for nonlinear systems under the condition of large-signal input [13–15]. Therefore, it is necessary to carry out a nonlinear analysis of PLLs. The existing literature seldom investigates high-order nonlinear systems and intelligent power control systems.

A SOGI is introduced into the PLL based on the linear Kalman filter to establish an intelligent aviation variable frequency power supply control system. The central angular frequency of the SOGI is obtained by the PLL feedback of the linear Kalman filter. Because the SOGI has infinite gain at its central angular frequency, it has a good filtering effect. The central angular frequency is a variable with time, constituting a high-order PLL system with strong nonlinearity. Then, the state equation of the system is derived and solved to obtain the stability region. The filter is optimized using the Long and Short-term Memory (LSTM) network to improve the intelligence of the design method. Finally, the effectiveness of the PLL based on the linear Kalman filter with SOGI is verified by simulation and experiment. The research presented here is mainly divided into three parts. Section 1 introduces the research theories and methods and leads to the problems to be solved. Section 2 designs the technique to improve the system’s stability and optimizes the parameters of the model to enhance the algorithm’s effectiveness. Section 3 tests this method to verify this method’s effectiveness in dealing with the related problems.

## 2 PLL structure of linear Kalman filter with SOGI

Due to the high harmonic content of aviation variable frequency power supply, the phase angle output by PLL contains high-frequency components. Thus, it is impossible to obtain the phase information of power supply voltage accurately. Especially for the grid-connected device based on a power electronic converter, synchronizing with the grid voltage is essential for regular operation. If the rectifier cannot accurately obtain the phase information of grid voltage, the power factor cannot be corrected, resulting in the injection of reactive power into the grid. Therefore, it is necessary to accurately obtain the phase information of power supply voltage under non-ideal conditions such as the long harmonic content of aviation variable frequency power supply. The fundamental frequency of aviation variable frequency power supply changes linearly, ranging 360Hz-800Hz. Consequently, the high-order harmonic frequency changes at a higher rate, increasing the difficulty of filter design. Therefore, designing an appropriate filter combined with PLL is essential to solve the phase-locked problem when there are many harmonics in the aviation variable frequency power supply.

The aviation power distribution technology gradually develops from manual centralized control to computer control and turns to the intelligent control field [16]. The research on the control of aviation variable frequency power supply is a vital basis to ensure the safety of aviation power systems. This paper uses the linear Kalman filter as the PLL filter. Besides, good filtering results are achieved with the help of the wireless gain effect of the SOGI. The central angular frequency of the SOGI is returned by the output angular frequency *ω*_*g*_ of the Kalman filter PLL. Fig 1 displays the PLL structure. The stability of the working frequency is ensured by polyphase control of the input current. The structure of Kalman filter PLL is given in reference [13], as shown in Fig 2. This is an optimized structure based on Fig 1 to avoid the influence of loop instability and phase noise on the equipment.

**Fig 1:** Structure of PLL.

**Fig 2:** PLL structure of the linear Kalman filter.

### 2.1 PLL structure based on the linear Kalman filter optimized by the neural network

PLL is a device used to generate clock signals, which needs incredibly high performance. In the process of oscillation control, the equipment is required to have a high-frequency coverage to avoid the influence of loop instability and phase noise on the equipment. The structure of the LSTM network is obtained after optimization based on a cyclic neural network. Each neuron in the network has a set of independent parameters. However, there is a connection relationship between neurons, which can preserve the potential relationship in the data for a long time and positively affect processing time series problems [17]. Therefore, the LSTM network is suitable for processing important events with relatively long intervals and delays in time series.

Here, the LSTM network is employed to optimize the Kalman filter PLL. According to Fig 2, the time-domain equation between the phase angle *θ*_*g*_ and angular frequency *ω*_*g*_ output by the Kalman filter PLL, and the three-phase grid voltage *v*_*a*_, *v*_*b*_ and *v*_*c*_ after synchronous coordinate transformation can be expressed by Eq (1).


$$\left\{ \begin{array}{l} \omega_{g}=\int (k_{2}v_{q}+\int k_{1}v_{q}dt)dt\\ \theta_{g}=\int (\omega_{g}+k_{3}v_{q}-\frac{T_{s}}{2}\int k_{1}v_{q}dt)dt \end{array}\right.$$ (1)

In Eq (1), *k*_*1*_, *k*_*2*_, and *k*_*3*_ are coefficients, and *T*_*s*_ represents the sampling period.

Fig 3 illustrates the structure of the neural network. The neural network includes three layers: the input layer, hidden layer, and output layer, through which the data is input and processed. The linear Kalman filter PLL based on LSTM is multi-configuration. The interior neural network module takes the input signal as training and outputs the digital signal of control voltage to control the voltage passing through PLL.

**Fig 3:** Neural network structure.

### 2.2 Structure of SOGI

SOGI is a second-order integrator and an integral part of the controller. However, SOGI is easy to oscillate and has poor stability at the characteristic frequency point. Hence, SOGI with damping is used instead, which has the characteristics of frequency selection and low-pass filtering to suppress harmonics and achieve synchronization and orthogonal with the input signal. Fig 4 shows the structure of SOGI, where the center angular frequency is obtained by the output angular frequency *ω*_*g*_ of Kalman filter PLL. The time-domain equation of SOGI is expressed by Eq (2).


$$\left\{ \begin{array}{l} v^{'}=\int [(v-v^{'})k-qv^{'})\omega^{'}dt\\ qv^{'}=\omega^{'}\int v^{'}dt\\ \omega^{'}=\omega_{g} \end{array}\right.$$ (2)

**Fig 4:** Structure of SOGI.

In Eq (2), *k* denotes the damping coefficient of SOGI, *v*`stands for the grid voltage, and *ω`*refers to the angular frequency.

## 3 System stability analysis and parameter design

According to Fig 1, the real-time angular frequency output by the system is fed back to SOGI. Because the frequency of aviation variable frequency power supply changes in real time, the whole system constitutes a high-order nonlinear structure [18].

Since _*Vα*_ and *v*_*β*_ are linear transformation of three-phase input voltage *v*_*a*_, *v*_*b*_, and *v*_*c*_, they can be regarded as the input of the system. According to Fig 1 and Eq (2), there are:

$$v_{\alpha }^{'}=\int \left[k(v_{\alpha }-v_{\alpha }^{'})-qv_{\alpha }^{'}\right]\omega_{g}dt$$ (3)

$$qv_{\alpha }^{'}=\omega_{g}\int v_{\alpha }^{'}dt$$ (4)

$$v_{\beta }^{'}=\int \left[k(v_{\beta }-v_{\beta }^{'})-qv_{\beta }^{'}\right]\omega_{g}dt$$ (5)

$$qv_{\beta }^{'}=\omega_{g}\int v_{\beta }^{'}dt$$ (6)

According to the transformation formula from *αβ* axis to *dq* axis, the relationship between the system output phase angle and each quantity can be presented as Eq (7).


$$v_{q}=(v_{\beta }^{'}+qv_{\alpha }^{'})\cos\theta_{g}-(v_{\alpha }^{'}-qv_{\beta }^{'})\sin\theta_{g}$$ (7)

Therefore, from Eq (1) and Eqs (3) ~ (7), the time domain equation of the whole system can be expressed as Eq (8).


$$\left\{ \begin{array}{l} v_{\alpha }^{'}=\int \left[k(v_{\alpha }-v_{\alpha }^{'})-qv_{\alpha }^{'}\right]\omega_{g}dt\\ qv_{\alpha }^{'}=\omega_{g}\int v_{\alpha }^{'}dt\\ v_{\beta }^{'}=\int \left[k(v_{\beta }-v_{\beta }^{'})-qv_{\beta }^{'}\right]\omega_{g}dt\\ qv_{\beta }^{'}=\omega_{g}\int v_{\beta }^{'}dt\\ v_{q}=(v_{\beta }^{'}+qv_{\alpha }^{'})\cos\theta_{g}-(v_{\alpha }^{'}-qv_{\beta }^{'})\sin\theta_{g}\\ \omega_{g}=\int (k_{2}v_{q}+\int k_{1}v_{q}dt)dt\\ \theta_{g}=\int (\omega_{g}+k_{3}v_{q}-\frac{T_{s}}{2}\int k_{1}v_{q}dt)dt \end{array}\right.$$ (8)

Then, state variables are selected as follows:

$$\left\{ \begin{array}{l} x_{1}=v_{\alpha }^{'}\\ x_{2}=\frac{qv_{\alpha }^{'}}{\omega_{g}}\\ x_{3}=v_{\beta }^{'}\\ x_{4}=\frac{qv_{\beta }^{'}}{\omega_{g}}\\ x_{5}=\int v_{q}dt\\ x_{6}=\omega_{g}\\ x_{7}=\theta_{g} \end{array}\right.$$ (9)

Eq (8) is transformed into an equation of state as shown in Eq (10).


$$\left\{ \begin{array}{l} {\dot{x}}_{1}=kv_{\alpha }x_{6}-kx_{1}x_{6}-x_{2}x_{6}^{2}\\ {\dot{x}}_{2}=x_{1}\\ {\dot{x}}_{3}=kv_{\beta }x_{6}-kx_{3}x_{6}-x_{4}x_{6}^{2}\\ {\dot{x}}_{4}=x_{3}\\ {\dot{x}}_{5}=(x_{3}+x_{2}x_{6})\cos x_{7}-(x_{1}-x_{4}x_{6})\sin x_{7}\\ {\dot{x}}_{6}=k_{2}(x_{3}+x_{2}x_{6})\cos x_{7}-k_{2}(x_{1}-x_{4}x_{6})\sin x_{7}+k_{1}x_{5}\\ {\dot{x}}_{7}=x_{6}+k_{3}(x_{3}+x_{2}x_{6})\cos x_{7}-k_{3}(x_{1}-x_{4}x_{6})\sin x_{7}-\frac{T_{s}}{2}k_{1}x_{5} \end{array}\right.$$ (10)

According to Eq (10), this system is a seventh order nonlinear system, and the stability of the system is determined by parameters *k*, *k*_*1*_, *k*_*2*_, *k*_*3*_, and *T*_*s*_. Therefore, the values of *k*_*1*_, *k*_*2*_, *k*_*3*_, and *T*_*s*_ are first determined to select the bandwidth of Kalman filter PLL, and then, the value of *k* is decided to ensure the stability of the system [19].

Fig 5 illustrates the small signal model [13] of linear Kalman filter PLL. Then, the closed-loop transfer function of the linear Kalman filter PLL can be written as Eq (11).


$$G(s)=\frac{{\tilde{\omega }}_{g}(s)}{\omega_{g}(s)}=\frac{k_{2}s+k_{1}}{s^{3}+k_{3}s^{2}+k_{2}s+k_{1}}$$ (11)

**Fig 5:** Small signal model of the linear PLL based on Kalman filter.

To ensure the stability of the PLL system of linear Kalman filter, the root of the characteristic equation of its closed-loop transfer function is set as a negative real root and a pair of negative real part conjugate roots, as shown in Eq (12).


$$s_{0}=-w_{n}R,s_{1,2}=-w_{n}Exp(\pm j\phi )$$ (12)

In Eq (12), *w*_*n*_>0, *R*>0, and $0<\phi <\frac{\pi }{2}$.

Substituting Eq (12) into the characteristic equation, there is:

$$k_{1}=Rw_{n}^{3},k_{2}=(1+2R\cos\phi )w_{n}^{2},k_{3}=(R+2\cos\phi )w_{n}$$ (13)

Substituting Eq (13) into Eq (11), Eq (11) can be expressed as:

$$G(s)=\frac{(1+2R\cos\phi )w_{n}^{2}s+Rw_{n}^{3}}{s^{3}+(R+2\cos\phi )w_{n}s^{2}+(1+2R\cos\phi )w_{n}^{2}s+Rw_{n}^{3}}$$ (14)

The bandwidth *f*_*b*_ of PLL of linear Kalman filter is determined by parameters *R*, *w*_*n*_, and *ϕ*.

According to the definition of bandwidth, *G* represents the bandwidth. Then, there is:

$$20\mathrm{lg}|G(j2\pi f_{b})|=20\mathrm{lg}|G(j0)|-20\mathrm{lg}\sqrt{2}$$ (15)

Then, the relationship between bandwidth and various parameters is:

$$\frac{w_{n}^{2}\sqrt{R^{2}w_{n}^{2}+{\left(2R\cos\phi +1\right)}^{2}{\left(2\pi f_{b}\right)}^{2}}}{\sqrt{{\left({\left(2\pi f_{b}\right)}^{2}-w_{n}^{2}\right)}^{2}+4w_{n}^{2}\cos^{2}\phi {\left(2\pi f_{b}\right)}^{2}}\sqrt{R^{2}w_{n}^{2}+{\left(2\pi f_{b}\right)}^{2}}}=\frac{1}{\sqrt{2}}$$ (16)

Through reference [7], the change of parameter *w*_*n*_ has a great impact on the bandwidth. Therefore, let *R* = 1, and *ϕ* = π/3, and *f*_*b*_ is determined by the parameter *w*_*n*_. The bandwidth is set as 100Hz, 200Hz, and 300Hz, respectively, and the values of parameter *w*_*n*_ are summarized in Table 1 [20].

**Table 1:** Values of *w*_*n*_ in different bandwidths.

*R* = 1*ϕ* = π/3	*f*_*b*_ = 100Hz	*f*_*b*_ = 200Hz	*f*_*b*_ = 300Hz
*w*_*n*_	369.478	738.955	1108.433

Firstly, the bandwidth of PLL based on linear Kalman filter is selected. Then, the filtering performance and dynamic performance of the PLL based on linear Kalman filter under three different bandwidths are compared after adding a SOGI.

Eq (17) represents A phase voltage in the three-phase balanced power grid system.


$$v_{a}=115\sqrt{2}\cos\omega t+15\cos(5\omega t+18^{\circ })+8\cos(7\omega t+15^{\circ })+5\cos(11\omega t+12^{\circ })$$ (17)

The fundamental wave frequency is set to 400Hz, the fundamental voltage of *v*_*a*_ is expressed as *v*_*afund*_, and the effective value is 115V. Besides, the total voltage distortion rate is 10.8%, the maximum single voltage distortion rate is 9.2%, and the parameter of SOGI is 1. The simulation results of linear Kalman filter under the above three bandwidths are compared.

As shown in Fig 6, the angular frequency *ω*_*g*_ output by PLL can reach the steady-state value of 800πrad/s under three bandwidths. Moreover, the dynamic response of the bandwidth at 300Hz is better, but the oscillation time is longer before entering a steady state. The bandwidth has the slowest dynamic response at 100Hz.

**Fig 6:** Simulation results of *ω*_*g*_ under three bandwidths.

Fig 7 displays the comparison results of cos*θ*_*g*_ output by PLL after 100 times expansion with *v*_*a*_ and *v*_*afund*_. Under these three bandwidths, the phase-locked accuracy is high. The Total Harmonic Distortion (THD) of cos*θ*_*g*_ output by PLL under the three bandwidths are 0.97%, 0.98%, and 1.01%, respectively, showing a brilliant filtering effect.

**Fig 7:** Simulation results of cos*θ*_*g*_ under three bandwidths.

Considering both the dynamic response and filtering effect of PLL, PLL has the best effect when the bandwidth of PLL based on linear Kalman filter is 200Hz.

The PLL bandwidth of linear Kalman filter is set to 200Hz, so the corresponding parameters are *R* = 1, *ϕ* = π/3, and *w*_*n*_ = 738.955.

- *f*_*b*_ = 100Hz
- *f*_*b*_ = 200Hz
- *f*_*b*_ = 300Hz

According to Eq (13), *k*_1_ = 738.955^3^, *k*_2_ = 1,092,108.98,405, and *k*_3_ = 1,477.91.

In reference [12], the solution of differential equations is used to judge the stability of the system. Since the stability of the system is independent of the input, let *v*_*α*_ = 1V, *v*_*β*_ = 1V, and the sampling period *T*_*s*_ *=* 0.000,125s. In addition, the ode23tb function of MATLAB is utilized to solve the solution of differential equations. Fig 8 provides the solutions of the differential equations when the parameter *k* of SOGI takes different values.

- *k* = 0.5
- *k* = 1
- *k* = 2
- *k* = 3
- *k* = 5

**Fig 8:** Solutions of differential equations under different values of *k*.

From Fig 8, when *k* = 0.5, *k* = 1, *k* = 2, *k* = 3, and *k* = 5, *x*_*1*_ ~ *x*_*6*_ converge with the change of time, while *x*_*7*_ is divergent. However, *x*_*7*_ = *θ*_*g*_ is the quantity varying with time, and *x*_*5*_ = 0. Therefore, *v*_*q*_ is a bounded quantity and an error quantity, so the system is stable. Since the stability region of the system is a sufficient condition for the stability of the system, a conservative stability region can be selected, and *k* is stable in [0.5, 3].

## 4 Simulation and experimental verification

It is concluded in the previous section that the system parameters *k*_*1*_ = 738.955^3^, *k*_*2*_ = 1,092,108.98405, *k*_*3*_ = 1,477.91, *T*_*s*_ = 0.000,125s, and *k* is stable in the range of [0.5, 3]. Then, Simulink is for simulation.

In the three-phase balanced power grid system, the A phase voltage is represented by Eq (17), the fundamental wave frequency is 360 Hz ~ 800 Hz, and the change rate is a linear change of 200 Hz/s according to the DO—160G standard.

Fig 9 illustrates the simulation waveform of angular frequency *ω*_*g*_ and phase angle *θ*_*g*_ when *k* = 0.5, *k* = 1, *k* = 2, *k* = 3, and *k* = 5, respectively.

(1) *ω*_*g*_
(2) *θ*_*g*_
  (a) *k* = 0.5
(1) *ω*_*g*_
(2) *θ*_*g*_
  (b) *k* = 1
(1) *ω*_*g*_
(2) *θ*_*g*_
  (c) *k* = 2
(1) *ω*_*g*_
(2) *θ*_*g*_
  (d) *k* = 3

**Fig 9:** Simulation under frequency conversion.

From the above waveforms, when *k* = 0.5, *k* = 1, *k* = 2, *k* = 3, and *k* = 5, the angular frequency *ω*_*g*_ output by PLL finally changes linearly with the change rate of 400πrad/s^2^, and the output phase angle *θ*_*g*_ also reaches a stable state. Therefore, *k* is proved to be stable within [0.5, 3]. Through Fig 8, when *k* is in the range of [0.5, 3], the output phase angle linearity is good, and the angular frequency is stable. Therefore, *k* in the range of [0.1, 3] can meet the phase-lock requirements.

Then, the output phase angle *θ*_*g*_ of the PLL based on Kalman filter with SOGI is compared with that of the PLL based on Kalman filter without SOGI under the same input power supply. Fig 10 reveals the results when *k* = 1, where A refers to the curve of Kalman filter with SOGI, and B stands for the curve of Kalman filter without SOGI.

**Fig 10:** Comparison of simulation results of *θ*_*g*_.

Fig 10 indicates that the phase angle linearity of the output of the PLL based on Kalman filter with SOGI is obviously better, and the high-frequency components in the phase angle are filtered out.

Furthermore, the anti-interference energy of PLL is verified when the grid voltage is unbalanced. In this test, *k* = 1, the power supply voltage is shown as Eq (17), the fundamental frequency is 360 Hz ~ 800, and the linear change rate is 200 Hz/s. Besides, the fundamental voltage of C phase suddenly changes to 0 at 0.1s. Then, cos*θ*_*g*_ output by PLL after 100 times expansion is compared with *v*_*afund*_. Fig 11 illustrates the simulation results under the condition of power grid voltage imbalance.

**Fig 11:** Simulation results of cos*θ*_*g*_ under unbalanced grid voltage.

It can be seen from Fig 11 that after the fundamental voltage of C phase suddenly changes to 0, the phase-lock accuracy is restored for about one cycle. This result proves that it has good anti-interference ability.

Neural networks with different amounts of layers are compared to verify the effect of the neural network on phase-lock. Fig 12 shows the comparison results of convolutional neural network (CNN) and LSTM network.

**Fig 12:** Comparison results of different networks.

As can be seen from the results in Fig 12, the accuracy of the CNN algorithm is 75% at the highest and 70% at the lowest. The highest accuracy of the LSTM algorithm is 80%, and the lowest is 75.5%. Therefore, with different hidden layers, the LSTM network has better performance than CNN, and the highest accuracy can reach about 80%. Compared with similar research, the method designed here realizes the intelligent aviation power frequency conversion control method, with specific practical value.

## 5 Discussion

The PLL based on linear Kalman filter is combined SOGI with to establish the intelligent phase-locked technology of aviation variable frequency power supply. For the high-order phase-locked loop system with strong nonlinearity, the state equations of the whole phase-locked loop are derived and solved to obtain a stable region of the system. The filter is optimized based on the LSTM network. The results show that in the three-phase balanced power grid system, *k* ranging [0.1, 3] can meet the phase-locked requirement. The output phase angle linearity of Kalman filter PLL with SOGI is obviously better than that under the above same input power supply, and the high-frequency component in the phase angle is filtered out. The experimental results indicate that the addition of LSTM network can realize the intelligent aviation power frequency conversion control. Therefore, this paper can achieve the accurate phase-locked of aviation variable frequency power supply.

## 6 Conclusion

The PLL based on linear Kalman filter and SOGI can adapt to wide input frequency and has the advantages of high phase-locked accuracy and fast dynamic response. Still, its phase-locked accuracy is affected by power supply voltage distortion. This method is simulated and verified in the stability region by designing the experiment. It is proved that the linear Kalman filter PLL with SOGI can solve the problem that the output phase angle contains high-frequency components when the distortion rate is 10%. The accuracy of the optimized model is more than 80%. Therefore, this PLL method has a strong anti-interference ability under the condition of power grid voltage imbalance, which is conducive to the realization of accurate phase-locked. Compared with similar studies, the method proposed here can control the aviation variable frequency power supply more intelligently and effectively improve the power supply stability of the aviation power supply system. This paper provides a reference for the application of related technologies. However, there are some deficiencies in the current research. For example, the neural network excessively depends on data sets, but there are few types of data set labels, which cannot well simulate the situation in the actual environment. Moreover, the practical application effect of the designed method also needs to be further optimized. Therefore, the follow-up research will further explore the designed algorithm and its practical application.

## Supporting information

S1 Data (XLSX)
